# Lightweight YOLOv4 with Multiple Receptive Fields for Detection of Pulmonary Tuberculosis

**DOI:** 10.1155/2022/9465646

**Published:** 2022-03-31

**Authors:** Zhitao Guo, Jiahao Wang, Jinghua Wang, Jinli Yuan

**Affiliations:** College of Electronic Information Engineering, Hebei University of Technology, Tianjin 300401, China

## Abstract

The characteristics of pulmonary *tuberculosis* are complex, and the cost of manual screening is high. The detection model based on convolutional neural network is an essential method for assisted diagnosis with artificial intelligence. However, it also has the disadvantages of complex structure and a large number of parameters, and the detection accuracy needs to be further improved. Therefore, an improved lightweight YOLOv4 pulmonary *tuberculosis* detection model named MIP-MY is proposed. Firstly, over 300 actual cases are selected to make a common dataset by professional physicians, which is used to evaluate the performance of the model. Subsequently, by introducing the inverted residual channel attention and the pyramid pooling module, a new structure of MIP is created and used as the backbone extractor of MIP-MY, which could further decrease the number of parameters and fuse context information. Then the multiple receptive field module is added after the three effective feature layers of the backbone extractor, which effectively enhances the information extraction ability of the deep feature layer and reduces the miss detection rate of small pulmonary *tuberculosis* lesions. Finally, the pulmonary *tuberculosis* detection model MIP-MY with lightweight and multiple receptive field characteristics is constructed by combining each improved modules with multiscale structure. Compared to the original YOLOv4, the model parameters of MIP-MY is reduced by 47%, while the mAP value is raised to 95.32% and the miss detection rate is decreased to 6%. It is verified that the model can effectively assist radiologists in the diagnosis of pulmonary *tuberculosis*.

## 1. Introduction

Pulmonary *tuberculosis* has become a global public health emergency, in which people are infected with a chronic infectious disease caused by *Mycobacterium tuberculosis* [1]. According to the World Health Organization (WHO) survey, pulmonary *tuberculosis* is one of the leading causes of death from infectious diseases around the world. It is estimated that about 64% of 10 million pulmonary *tuberculosis* cases are detected and treated each year [2]. Improving the awareness rate and early detection rate of pulmonary *tuberculosis* plays a vital role in the treatment of the disease, as well as the prevention of the spread of the disease [3]. Computed tomography (CT) is one of the auxiliary imaging diagnostic methods for *tuberculosis* screening, having a lower missed detection and false detection rate than chest radiographs. It is a more efficient choice to adopt CT technology to identify substantial chest lesions and detect the severity of lung diseases in patients with *tuberculosis* [4].

With the development of artificial intelligence, some scholars have gradually begin to integrate the deep learning image processing algorithm of deep learning with CT technology to achieve a more accurate diagnosis and detection of lung diseases. Many deep learning models of computer-aided diagnosis have been built based on the deep convolution neural network (DCNN). Gao et al. [5] combined with CT technology proposed a high-precision classification model of five types of pulmonary *tuberculosis* based on CNN and support vector machine. Ma et al. [6] proposed an automatic detection model of active pulmonary *tuberculosis* based on U-Net [7], which can detect the location of lesions more accurately. Liu et al. [8] built simulated and real data sets based on CT images of lung cancer lung nodules and realized automatic detection of lesions through an improved single-stage target detection network YOLOv3 [9]. Yang et al. [10] took the two-stage target detection network Faster-RCNN as the main body, which improved the detection accuracy of pulmonary *tuberculosis*. However, its parameter scale was large and was not conducive to generalization.

Considering that the current detection model for pulmonary CT disease has the problem of excessive parameters and does not use effective lightweight methods, it may be a feasible strategy to learn from the lightweight methods in other detection fields. In reference [11], Ye et al. [11] replaced the backbone network of YOLOv4 [12] through MobileNetv3 [13] and realized the lightweight of the model. Although Mobilenetv3 reduces the amount of parameters, if it is directly used in the detection of pulmonary *tuberculosis* CT, it may lack the mining of deep feature information of the image, which is not enough to solve the problem of missed detection rate of small targets by YOLOv4, and the detection accuracy needs to be further improved. Reference [14] achieves lightweight by reducing the number of convolution layers in YOLOv5 [15], which obviously improves the detection speed. However, because the lightweight YOLOv5 focuses on the detection of large targets, the detection performance of small targets is still slightly insufficient. Small lesions on pulmonary *tuberculosis* CT cannot be ignored. The structure and performance of YOLOv5 are less different from those of YOLOv4. Therefore, improving on YOLOv4 is an effective strategy. CT images of pulmonary *tuberculosis* have mainly have typical features such as cavity [16] and tree-in-bud pattern [17]. However, open data sets are uneven and there is no uniform format, so it is essential to design a set of standard datasets. Additionally, the existing *tuberculosis* detection model has a large number of parameters and consumes a lot of computing resources, which makes it difficult to be applied to medical institutions with a large number of high-performance equipment. Therefore, it is an important goal to realize the lightweight of the model. At the same time, an ordinary lightweight detection model cannot obtain the deeper semantic information of CT images, resulting in a high rate of missed detection. Therefore, ensuring high detection accuracy and efficiency of *tuberculosis* simultaneously is one of the main objectives of this study, which is of great significance for *tuberculosis* screening and diagnosis.

The major contributions in our study can be summarized as follows.

1. At present, some existing models lack the ability to distinguish small objects, so that the miss detection rate stays in a high position without going down. For this reason, a new module of the multiple receptive field block (MRFB) with dilated convolution is designed in this paper. This module expands the acceptance range of the pulmonary *tuberculosis* detection model. It enhances the ability of feature extraction for various sizes of lesions to prevent some small size lesions that are detrimental to identify from being omitted.
2. Location, classification, and the confidence score of pulmonary *tuberculosis* lesions are equally important factors affecting the detection capability of the model. Taking these three factors as optimization objects can further improve the detection accuracy of the model. Consequently, an integrated loss function is designed which can train these three factors simultaneously. In the iterative training process of the model, the actual location of the lesions will be continuously updated continuously by the integrating loss function, the classification of the lesions will be determined, and the reliability of all lesions will be optimized simultaneously.
3. Lightweight convolution layers are constructed to reduce the number of model parameters, and a new backbone extractor MIP is designed. Its internal inverted residual channel attention module and pyramidal pooling layer can assist the model in extracting the deeper semantic information of pulmonary *tuberculosis* lesions. It realizes lightweight in structure and avoids overfitting to a certain extent, enhances the relationship between the different sizes of regions on feature maps, and completes the fusion of multiscale feature information.

The remainder of this paper is organized as follows. In Section 1, a standard data set of pulmonary *tuberculosis* is built, which contains CT slices of 300 patients with pulmonary *tuberculosis*. And a lightweight method is also introduced that is used in the pulmonary *tuberculosis* detection model. In Section 2, a pulmonary *tuberculosis* detection model MIP-MY is designed based on an improved YOLOv4 algorithm. In section 3, we carry out a quantitative analysis and score comparison on the results of networks. Finally, we discuss some related issues and make conclusions in Section 4.

## 2. Dataset and Lightweight Method

Currently, the public data set on CT of pulmonary *tuberculosis* CT is scarce, with incomplete image data, and the format is not unified. Therefore, it is imperative to design a standard data set for the research of this study. The lightweight detection model is one of the targets to be achieved in this paper. While completing the lightweight, we must ensure a higher accuracy, which is also the difficulty in designing the pulmonary tuberculosis detection model.

### 2.1. Creation of Dataset

The experimental data for this study is the actual data set provided by the Imaging Department of Beijing Chest Hospital, China. A total of 300 CT cases of pulmonary *tuberculosis* are collected to form the experimental data set. Each CT slice is segmented according to the thickness standard of 1.25 mm, of the which the CT sections of pulmonary *tuberculosis* cavity and the tree-in-bud pattern accounted for 50%, respectively. The cavity diameter in the data set ranges from 10 mm to 126.4 mm, and the tree-in-bud pattern with uniform density is selected as the sample. The areas from 16 × 16 to 128 × 128 on the CT slices are defined as a cluster of tree-in-bud pattern lesions, respectively. The distribution maps of the size of the lesions size in the dataset are shown in Figure 1. As shown from Figures 1(a) and 1(b), there are more small cavities with a diameter less than or equal to 30 mm, accounting for about 33% of the total. And more samples of tree-in-bud patterns in clusters with the size from 32 × 32 to 64 × 64 account for about 40% of the total. The standard for the above data set was established by three clinical doctors with more than five years of experience at Beijing Chest Hospital after discussion at the meeting, and the LabelImg tool [18] tool was used to outline and calibrate the lesion of pulmonary *tuberculosis*, providing a guarantee of the consistency and validity of the dataset.

The unified preprocessing of each CT image is carried out, and its format is converted from DICOM to PNG, which is more convenient for processing. The resolution is adjusted to 512 × 512, and the number of coding bits is 24. Additionally, to reduce interference to the detection model, background information is filtered, including bed board and clothing outside the outline of the lung.

The data set contains a total of 3764 CT slices of cavity and tree-in-bud pattern, from which 70% are randomly selected as the train set, the remaining 10% as test set 1, and the last 20% as test set 2. Test Set 1 is responsible for subsequent ablation experiments, while test set 2 is responsible for evaluating the diagnostic level of the pulmonary *tuberculosis* detection model.

Data enhancement enriches the diversity of the data set. Specifically, each CT image of the train set has a 40% chance of scaling and flipping horizontally and randomly distorting the input image with an aspect ratio of 0.8 to 2.0. These measures double the number of samples in the train set. This study has signed a patient information confidentiality agreement with the Imaging Department of Beijing Chest Hospital to filter out patients' sensitive information by technical means, and the right to use the dataset is merely effective in this study.

### 2.2. Lightweight Method

At present, the detection model based on the convolutional neural network has some problems such as a large number of parameters and long training time, which requires high hardware computing capacity. Therefore, this paper will adopt a lightweight method to modify the model to make it suitable for general hardware devices.

MobileNetv3 is a lightweight neural network commonly used in image processing. It is based mainly on the principle of separable depthwise convolution [19] to achieve the lightweight target.

Compared with traditional convolution, depthwise separable convolution has fewer parameters. The Depthwise Separable Convolution traverses only one by one corresponding to the input channel and then expands the number of output channels by 1 × 1 Pointwise Convolution. The principle of Depthwise Separable Convolution is shown in Figure 2.

The number of parameters required for traditional convolution and Depthwise Separable Convolution is set to *N*_1_ and *N*_2_ respectively, and their calculation formulas are shown in formulas (1) and (2).

(1) $$\begin{array}{c} N_{1}=i_{h}\cdot i_{w}\cdot c_{\text{in}}\cdot c_{\text{out}}\cdot k^{2}, \end{array}$$

(2) $$\begin{array}{c} N_{2}=i_{h}\cdot i_{w}\cdot c_{\text{in}}\cdot \left(k^{2}+c_{\text{out}}\right), \end{array}$$

where *i*_*h*_ and *i*_*w*_ are the height and width of the input tensor, *k* is the size of the selected convolution kernel, and *c*_in_ and *c*_out_ respectively represent the number of input and output channels. Furthermore, as shown in formula (3)

(3) $$\begin{array}{c} \frac{N_{1}}{N_{2}}=\frac{k^{2}\cdot c_{\text{out}}}{k^{2}+c_{\text{out}}}. \end{array}$$

In practical application, *N*_2_ is much less than *N*_1_, which means Depthwise Separable Convolution can reduce computational overhead to a greater extent.

The model in reference [11] replaced YOLOv4's backbone extractor CSPDarkNet53 [20] by MobileNetv3, which reduces the number of parameters to a great extent. However, it is difficult to achieve high accuracy if this model is directly used to detect pulmonary *tuberculosis*. If the lightweight of the model is improved at the expense of detection accuracy, that will be contrary to the main target of our study. Therefore, this article will ameliorate the MobileNetv3 and YOLOv4 to reduce the parameters of the pulmonary *tuberculosis* detection model, improve detection efficiency as well as the accuracy.

## 3. Design of Pulmonary Tuberculosis Detection Model

The structure of the pulmonary *tuberculosis* detection model refers to the YOLOv4 method, and the structure of YOLOv4 is shown in Figure 3. As can be seen from Figure 3, the original YOLOv4 enhances the learning feature information ability by virtue of the CSPDarkNet53 as the backbone part, which reduces model overfitting through the combination of traditional convolution and residuals. The neck part is spliced with SPP module (spatial pyramid pooling) [21] and PAN module (path aggregation network) [22] to complete the multiscale feature information fusion of different regions. Finally, the multiscale feature information is collected by using the three Heads in the prediction part to generate the final prediction bounding box. The original YOLOv4 focuses on efficiency and accuracy, but has not yet achieved satisfactory results in the field of pulmonary *tuberculosis* detection.

Different from the original YOLOv4, the developed pulmonary *tuberculosis* detection model named MIP-MY comprises three parts: a backbone extractor, enhanced feature extractor, and a bounding box generator. A new backbone extractor MIP is designed for MIP-MY, which is the lightweight module of the detection model. MIP uses the newly designed IRCA (Inverted Residual Channel Attention) module and pyramid pooling module to achieve lightweight. MIP can extract abundant contextual information and make preliminary sampling for pulmonary *tuberculosis*. Then, in order to capture lesions of different sizes, we designed MRFB (multiple accept field block) module to construct the enhanced feature extractor, which can have a wider acceptance field to reduce the missed detection of small lesions. According to the momentous information (lesion location, classification, and confidence score) output by the bounding box generator, a comprehensive loss function is designed to regression the lesion location and optimize the confidence score.

### 3.1. Backbone Extractor MIP

The function of the backbone feature extractor MIP is to analyze the CT images of pulmonary *tuberculosis* and extract the image features of pulmonary *tuberculosis* lesions. In this paper, according to the inverted residuals structure of MobileNetv3, a new IRCA (Inverted Residuals Channel Attention) module is constructed using channel attention mechanism. By virtue of the inverted residuals structure, this module can build a deeper network without a gradient explosion. An introduced channel attention mechanism can capture the corresponding context information on each IRCA module and improve the feature extraction ability of the network. The structure of IRCA is shown in Figure 4. As a significant part of MIP, IRCA module constructs seven effective feature layers for MIP to extract the lesions information of pulmonary *tuberculosis*. The MIP connects a pyramid pool module in the last effective feature layer to obtain multiple scale feature information. The structure of MIP and pyramid pooling module is shown in Figure 5.

Before completing the 1 × 1 Pointwise Convolution operation, the IRCA module carries out Global-Average pooling to obtain the feature graph with a smaller size, and calculate the weight of the feature map through Relu6 and Hard-Swish activation function. Finally, the weighted multiplication is performed through channel attention. The calculation formula of Global-Average pooling is shown in formula (4).

(4) $$\begin{array}{c} y_{\text{avg}}=\frac{\sum_{i=0}^{n}\sum_{j=0}^{n}x_{i,j}}{n^{2}}, \end{array}$$

where *x*_*i*,*j*_ is the pixel on the 2D slices of feature maps and *y*_avg_ is the pixel mean of the Global-Average pooling. The calculation formula of Relu6 and Hard-Swish activation function is shown in formulas (5) and (6).

(5) $$\begin{array}{c} f_{1}\left(y_{\text{avg}}\right)=\min\left(\max\left(0,y_{\text{avg}}\right),6\right), \end{array}$$

(6) $$\begin{array}{c} f_{2}\left(y_{\text{avg}}\right)=y_{\text{avg}}\cdot \frac{f_{1}\left(y_{\text{avg}}+3\right)}{6}, \end{array}$$

where *f*_1_(*y*_avg_) is the activation result of ReLu6, and the upper limit of this value is 6. *f*_2_(*y*_avg_) is the activation result of Hard-Swish. It is found that the accuracy of a neural network can be enhanced by using the hard-swish activation function in deeper convolution layers.

(7) $$\begin{array}{c} f_{3}=X\cdot f_{2}\left(f_{1}\left(y_{\text{avg}}\right)\right), \end{array}$$

where the output *X* of the “Depthwise Separable Convolution” in formula (7) is a characteristic graph composed of *n*^2^ pixels, and *f*_3_ is the weighted calculation result of the whole channel attention.

In order to enable the backbone extractor to acquire information about the lesions information of different scales, this design draws lessons from the structure of PSPNet (Pyramid Scene Parsing Network) [23] and designs a pyramid pooling module as the integrated pooling layer of the backbone extractor (max pooling + average pooling), which combines four pooled kernels of various scales (32 × 32, 16 × 16, 8 × 8 and 4 × 4) to further analyze the location, size and other information about the lesions.

In summary, this design is improved by using the IRCA module and pyramid pooling module to compose the structure of a new backbone extractor MIP.

### 3.2. Enhanced Feature Extractor Dominated by MRFB

The last three effective feature layers of the MIP backbone extractor MIP will export feature maps with the resolution of the original image of 1 to 8, 1 to 16, and 1 to 32, respectively, providing pixel information of different sizes of lesions in pulmonary *tuberculosis* for subsequently enhanced feature extractor.

The initially enhanced feature extractor of YOLOv4 is mainly composed of SPP module and PAN module. SPP will take the result of the last feature layer of the backbone extractor as input and divide the feature map into three subregions of different sizes (8 × 8, 4 × 4, and 2 × (2) for maximum pooling, collecting multiscale eigenvalues. The PAN is a reciprocating structure responsible for collecting the output of three effective feature layers of the backbone extractor to build a feature pyramid. Each effective feature layer integrates the sampling information of the other two layers to complete multiscale feature lesions.

Although the initially enhanced feature extractor uses a multiscale feature fusion method to collect image information, the utilization of multireceptive field information is far from enough, and it is easy to ignore the feature expression of small targets. Therefore, in this section, combining the ideas of expansion convolution and receptive field amplification [24], the MRFB module is designed to optimize the enhanced feature extractor of YOLOv4. The structure of MRFB is shown in Figure 6.

Combined with the structure of the MRFB module, it can see that the MRFB module adopts parallel expansion convolution, and expands and samples the receptive field of the feature map through the collocation of three expansion rates (dilated rate takes 1, 3 and 5) and three convolution kernels (size takes 1 × 1, 3 × 3, and 5 × 5), and adds residual shortcut to prevent the loss of feature information, and finally splices the sampling results of each convolution to fuse the information of multiple receptive fields. As shown in Figure 6, the MRFB module, as the probe of PAN, is connected with the backbone feature extractor MIP, which makes up for the deficiency of PAN feature map information collection.

### 3.3. Bounding Box Generator and Decoder

The function of the bounding box generator is to achieve regression of the information from the pulmonary *tuberculosis* lesion (lesion size, class, and location), which is composed of three decoupling heads and a decoder. Each head generates three bounding boxes of different sizes on the multiscale feature map sampled by PAN to surround the pulmonary tuberculosis lesion. The parameters of the bounding box include the coordinates of the center point coordinates, size, class of lesion, and confidence score. However, this parameter information cannot directly reflect the position of the final bounding box in the picture. The information of the bounding box needs to be further decoded by the decoder.

#### 3.3.1. Decoding of Bounding Box

The bounding box is decoded with Anchor. Anchor is a predefined bounding box on each feature point of the input image. The activation function for its decoding is shown in formula (8).

(8) $$\begin{array}{c} \sigma \left(t\right)=\frac{1}{1+e^{-t}}, \end{array}$$

where *t* represents the confidence score and category probability of the bounding box, and these two kinds of parameters are mapped to the range of [0,1] by function *σ*(*t*). The decoding definition of the center point coordinates (*C*_*x*_, *C*_*y*_) of the bounding box is shown in formulas (9) and (10).

(9) $$\begin{array}{c} C_{x}=\;\sigma \left(x_{\text{offset}}\right)+A_{x}, \end{array}$$

(10) $$\begin{array}{c} C_{y}=\;\sigma \left(y_{\text{offset}}\right)+A_{y}, \end{array}$$

where the coordinate offset (*x*_offset_ and *y*_offset_) from the center point of the prediction box is the coordinate offset and the coordinate offset is relative to the center point of the prediction box. (*A*_*x*_, *A*_*y*_) is the center point coordinate of the Anchor, and the center point coordinates (*C*_*x*_, *C*_*y*_) of the bounding box is obtained after decoding.

The decoding formulas for the height and width of the bounding box are shown in formulas (11) and (12).

(11) $$\begin{array}{c} H=e^{h}\cdot A_{H}, \end{array}$$

(12) $$\begin{array}{c} W=e^{w}\cdot A_{W}, \end{array}$$

where the *h* and *w* are the height and width of the bounding box before decoding, *A*_*H*_ and *A*_*W*_ are the height and width of Anchor, and the height *H* and width *W* of the decoded bounding box is calculated, respectively.

After decoding, the pulmonary *tuberculosis* lesions at the same position in the image will be surrounded by a large number of bounding boxes, so it is necessary to filter the redundant bounding boxes according to the Intersection of Union threshold (IOU) (usually set to 0.5), and then filter out these bounding boxes with the highest confidence score through the nonmaximum suppression algorithm [25]. The mathematical definition of the IOU is shown in formula (13).

(13) $$\begin{array}{c} \text{IOU}=\frac{\left|b\cap^{\;}b^{gt}\right|}{\left|b\cup^{\;}b^{gt}\right|}, \end{array}$$

where the denominator represents the intersection of the area of the bounding box *b* and the real box *b*^*gt*^, and the numerator represents the union. IOU reflects the similarity between the predicted results of the detection model and the ground truth.

#### 3.3.2. Integrated Loss Function

The integrated loss function of the pulmonary *tuberculosis* detection network is mainly composed of regression loss *L*_CIOU_, class loss *L*_Class_ and confidence loss *L*_Conf_.

The general loss function of the detection model is shown in formula (14).

(14) $$\begin{array}{c} L=L_{\text{CIOU}}+L_{\text{Confidence}}+L_{\text{Class}}. \end{array}$$

The mathematical expression of regression loss *L*_CIOU_ is shown in formula (15).

(15) $$\begin{array}{c} \left\{\begin{array}{c} v_{i,j}=\frac{4}{\pi^{2}}{\left(\tan^{-1}\frac{W_{i,j}^{gt}}{H_{i,j}^{gt}}-\;\tan^{-1}\frac{W_{i,j}}{H_{i,j}}\right)}^{2},\\ \alpha_{i,j}=\frac{v_{i,j}}{1-{\text{IOU}}_{i,j}+v_{i,j}},\\ L_{\text{CIOU}}=\sum_{i}^{S^{2}}\sum_{j}^{N}\left[1-{\text{IOU}}_{i,j}+\frac{\rho \left(b_{i,j},b_{i,j}^{gt}\right)}{d_{i,j}^{2}}+\alpha_{i,j}v_{i,j}\right], \end{array}\right.\; \end{array}$$

where the subscript (*i*, *j*) shows the serial number of the *j* bounding box on the pixel point in the feature map, *S* is the resolution size of the feature maps and *i* is the number of predicted bounding boxes on every feature map. *W*_*i*,*j*_^*gt*^ and *H*_*i*,*j*_^*gt*^ are the width and height of the corresponding ground truth, *α*_*i*,*j*_*v*_*i*,*j*_ is the penalty factor of *L*_CIOU_, and *ρ*(*b*_*i*,*j*_, *b*_*i*,*j*_^*gt*^) is the Euclidean distance between the center point of the predicted bounding box and the ground truth, and *d*_*i*,*j*_ represents the diagonal distance of the smallest enclosed area that can contain both the predicted bounding box and the ground truth. The definition of class loss is shown in formula (16).

(16) $$\begin{array}{c} L_{\text{Confidence}}=\sum_{i}^{S^{2}}\sum_{j}^{N}O_{i,j}\left[-\log\left(E_{i,j}\right)\right]+\lambda \sum_{i}^{S^{2}}\sum_{j}^{N}\left(1-O_{i,j}\right)\left[-\log\left(1-E_{i,j}\right)\right], \end{array}$$

where the *O*_*i*,*j*_ is a binary number to judge whether the pulmonary *tuberculosis* focus is in the predicted bounding box, and *E*_*i*,*j*_ represents the confidence of every pulmonary *tuberculosis* focus. *λ* sets as 1 when the IOU is greater than the threshold, otherwise takes 0. The class loss *L*_Class_ is defined in formula (17).

(17) $$\begin{array}{c} L_{\text{Class}}=\sum_{i}^{S^{2}}\sum_{j}^{N}O_{i,j}\sum_{c\in \text{Classes}}^{M}\left[P_{i}\left(c\right)\log\left(P_{i}{}^{gt}\left(c\right)\right)+\left(1-P_{i}\left(c\right)\right)\log\left(1-P_{i}{}^{gt}\left(c\right)\right)\right], \end{array}$$

where *M* is the number of classes, *P*_*i*_(*c*) is the class score of the detection network decision, and *P*_*i*_^*gt*^(*c*) represents class score of the ground truth.

By improving the structure of the pulmonary *tuberculosis* detection model and the selection of the loss function, the *tuberculosis* detection model developed in this paper is named MIP-MY (MobileNet with Inverted residuals and Pyramid pooling - Multiple receptive fields of YOLO). The model creates a lightweight trunk extractor MIP based on the basis of YOLOv4 and uses the MRFB module to replace the ordinary convolution layer that enhances the partial redundancy of the feature extractor, which only takes up less memory to enhance the ability to obtain multiple receptive field features. Finally, the integrated loss function is aimed at completing the regression and classification of pulmonary *tuberculosis* lesion information at the model training.

The overall structure of the improved pulmonary *tuberculosis* detection model MIP-MY is shown in Figure 7.

### 3.4. Evaluation Method

The evaluation of the pulmonary *tuberculosis* detection model is mainly determined by the number of parameters, detection time of per CT, Precision, Recall, miss detection rate, and mean Average Precision (mAP) [26]. The Precision *F*_*Pr*_ is as shown in formula (18).

(18) $$\begin{array}{c} F_{Pr}=\frac{\text{TP}}{\text{TP}+\text{FP}}, \end{array}$$

where TP is the true positive of the sample, FP is the false positive, and the sum of them is the prediction result of the model. The recall rate *F*_*Re*_ is shown in formula (19).

(19) $$\begin{array}{c} F_{Re}=\frac{\text{TP}}{\text{FP}+\text{FN}}, \end{array}$$

where the FN is false negative, and the sum of FP and FN is the total amount of the real box. In this study, the miss detection rate is mapped from the average miss detection rate of pulmonary *tuberculosis* CT in the test set 2 to the logarithmic space, and its mathematical definition is as shown in formula (20).

(20) $$\begin{array}{c} \left\{\begin{array}{c} mr_{i}=1-\frac{{\text{TP}}_{i}}{{\text{TP}}_{i}+{\text{FP}}_{i}},\\ F_{Lamr}=e^{1/Q\sum_{i=1}^{Q}\log\left(\max\left(mr_{i},\varepsilon \right)\right)}, \end{array}\right. \end{array}$$

where *mr*_*i*_ represents the miss rate of a single CT slice and *Q* represents the total number of CT slices. Besides, log(0) has no mathematical meaning, a smaller value *ε* is set to prevent the independent variable of the logarithmic function from being zero.

The IOU by a threshold of 0.5 is set to determine the TP and FP of the sample, and the P-R curve of the detection model is constructed with Precision and Recall as horizontal and vertical coordinates, respectively. The mAP is equal to the mean area under the P-R curve of all categories. The mathematical definition of the mAP is shown in formula (21), where *n* is the total number of categories.

(21) $$\begin{array}{c} m\text{AP}=\frac{\sum_{0}^{n}\int E_{pr}\cdot E_{red}\left(E_{re}\right)}{n}. \end{array}$$

## 4. Experimental Setting and Analysis

The operating system for this experiment is Windows 10, and the processors are Intel Core i7 and RTX 2060. Take PyCharm as the integrated development environment and utilize the deep learning framework of Keras based on Python3.8. To adapt to model training, the initial learning rate is set at 1.0 × 10–4. Adam optimizer and 1000 iterative training are also selected. Finally, the cosine annealing algorithm is used so that the pulmonary *tuberculosis* detection model can adaptively adjust the learning rate according to the number of iterations.

### 4.1. Ablation Experiment

For the sake of investigating the contribution of the integrated loss function and different components (MIP and MRFB) to improve the accuracy of detection model MIP-MY, we selected test set 1 to carry out two groups of ablation experiments.

The first group verifies the influence of different sub-losses (regression loss *L*_CIOU_, class loss *L*_Class_ and confidence loss *L*_Conf_) in the integrated loss function on the detection performance of the model, and then compares them with the traditional cross-entropy loss.

The quantitative comparison of performance on each loss function is shown in Table 1. Any single sub-loss can not optimize the detection accuracy of the model, and it is accompanied by a huge miss detection rate. Similarly, the combination of any two sub-losses has no obvious improvement on the detection accuracy and miss detection rate. The experimental results show that the coordinate location, class, and confidence score of pulmonary *tuberculosis* lesions are indispensable factors and only by combining these three seed losses can we effectively improve the overall performance of MIP-MY. Compared with traditional loss of the cross-entropy loss function, integrated loss can obtain better training results.

The second group verifies the effectiveness of the improved components in this paper, that is, we observe the effects of the addition and deletion of MIP module and MRFB module on the mAP, the number of parameters, miss detection rate and detection time. And compared with the lightweight model in reference [11].To facilitate differentiation, we named the lightweight model introduced by Model 1 in reference [11] as MobileNetv3-YOLOv4, the model that uses only MIP is called Model 2 and the model that uses only MRFB is called Model 3. MIP-MY integrates all the improved modules.

The results of the ablation experiment are shown in Table 2. From these data, it can be inferred that, compared with Model 1, the number of parameters of Model 2 is only increased by 0.93 M, but the mAP is increased by 2.64%, and the miss detection rate is reduced by 3%. Model 3 only uses MRFB to improve its mAP to 91.92%, but because it does not adopt the lightweight module MIP, the number of parameters is still high and with lower detection efficiency. MIP-MY combines the advantages of two improved modules to make the structure lightweight with the expansion of the receptive field feature mapping. Its mAP jumps to 95.59%, 9.73% higher than model 1, and the miss detection rate decreases by 10%. Meanwhile, the number of parameters decreases by 4.73 M, and the detection time of 1.07 s is shortened.

### 4.2. Comparative Experiment of Mainstream Models

Generally, the *tuberculosis* detection model is highly efficient, highly precise and low memory consumption and easy to apply to clinical diagnosis. To further verify the reliability of the MIP-MY model, we use the test set 2 to compare with several mainstream target detection models. The test set 2 contains 347 cavity samples and 539 tree-in-bud pattern samples. These CT samples are used to evaluate the performance of different detection models.

The P-R curve of the cavity of pulmonary *tuberculosis* cavity and the tree-in-bud pattern detected by different models is shown in Figure 8. As can be seen from the graph, compared to other mainstream detection models, the scope surrounded by the P-R curve of MIP-MY is the largest. Especially in Figure 8(b), the optimization effect of MIP-MY on the P-R curve for detecting the tree-in-bud pattern is the most obvious, indicating that this model is easier to capture the clustered tree-in-bud pattern.

Table 3 shows the evaluation results of different pulmonary *tuberculosis* detection models on test set 2. Through quantitative analysis, the performance of the single-stage detection model of YOLOv3 in reference [8] and YOLOv4 in reference [12] is not up to the mark. The reason is that there are many small cavities and clusters of tree-in-bud pattern in test set 2, which can easily be confused with normal bronchi in the lung region, resulting in a high rate of missed detection in both models. In contrast, the U-Net in reference [6] and the two-stage detection model Faster-RCNN in reference [10] have adequate mAP and low miss detection rate, but these two models have a large number of parameters, so they may not be suitable for equipment with general computing power, and the detection time is slightly longer, so it is difficult to achieve the requirements of high efficiency.

The MIP-MY model proposed in this paper has a remarkable performance in test set 2. Compared with the YOLOv4 model, the precision is increased by 5.22%, recall is increased by 4.47%, mAP is increased by 8.11%, the number of parameters is reduced by about 47%, and the error detection rate is reduced by 8%. Furthermore, MIP-MY also has a higher detection efficiency, the detection time of a single pulmonary *tuberculosis* image is shortened by 5.9 s compared to the Faster-RCNN.

From the numerical analysis of the evaluation results, MIP-MY can meet the target of high detection accuracy, and its model parameters take up less space, further reinforces the degree of lightweight.

In this paper, the pulmonary *tuberculosis* detection effect of the proposed MIP-MY model MIP-MY proposed needs to be shown more intuitively. The detection results of cavity in each model are shown in Figures 9 and 10, and the detection results of tree-in-bud pattern are shown in Figures 11 and 12. Ground Truth is the real label prescribed by the imaging doctors, the pulmonary *tuberculosis* cavity is marked as “cavity” in the bounding box, the tree-in-bud pattern is marked as “tree-in-bud” in the bounding box, and the corresponding confidence score is attached to the bounding boxes, which reflects the credibility of these lesions identity.

Through the analysis of the detection results of YOLOv3 and YOLOv4, it is found that the confidence score of YOLOv3 detection cavity and tree-in-bud pattern is low, which may be due to the underutilization of multiscale feature information by YOLOv3. Although YOLOv4 has a high confidence score, it fails to detect small lesions because the down sampling scale of the backbone extractor is too large and the spatial and pixel information of some small lesions is ignored in the layer-by-layer feature extraction. However, if the down sampling scale is reduced, the detection accuracy of other targets cannot be guaranteed. In Figure 10, it shows that U-Net makes miss detection in a tiny cavity, compared with the ability of Faster-RCNN to accurately capture cavities of various sizes. But in the example in Figure 12, U-Net and Faster-RCNN also omitted the detection in some inconspicuous tree-in-bud pattern.

MRFB module can effectively solve these problems of missed detection about lesions. MIP-MY was observed to capture small cavities and clusters of tree-in-bud patterns that are difficult to identify, indicating that the multiple-receptive field information collection ability of the MRFB module produces a marked effect and avoids the risk of small targets being missed. At the same time, the pulmonary *tuberculosis* lesion detected by MIP-MY has a high-level confidence score, which provides a reliable digital explanation for the automatic diagnosis ability of the detection model.

## 5. Conclusions

In this paper, a lightweight detection model MIP-MY with multiple receptive fields is developed for the automatic detection of pulmonary *tuberculosis*. Through ablation experiments, the contribution of MIP module in model lightweight is verified, and the superior performance of MRFB module and integrated loss function in improving model detection accuracy is also verified. Comparative experiments with other references show that MIP-MY has a lower number of parameters, better detection efficiency and accuracy, and its multiple receptive field characteristics strengthen the attention to small lesions and greatly reduce the possibility of misdetection. To sum up, the improved model MIP-MY achieves higher detection accuracy, realizes the automatic detection of pulmonary *tuberculosis* cavity and tree-in-bud pattern with lower calculation cost, and has excellent imaging diagnostic potential of pulmonary *tuberculosis*. In subsequent studies, more effective data enhancement techniques can be used to enrich the diversity of pulmonary *tuberculosis* CT data, such as generating game networks (GAN) to generate more samples. In addition, the generality of the model will be studied to make MIP-MY model suitable for the detection of common lung diseases, including lung cancer and pneumonia.

## Figures and Tables

**Figure 1:** Distribution maps of the size of the lesions size. (a) Distribution maps of the cavity. (b) Distribution maps of the tree-in-bud pattern.

**Figure 2:** Principle of depthwise separable convolution.

**Figure 3:** The structure of YOLOv4.

**Figure 4:** The structure of the IRCA module.

**Figure 5:** The structure of MIP and pyramid pooling module.

**Figure 6:** The structure of MRFB module.

**Figure 7:** The overall structure of MIP-MY (a) Backbone extractor MIP; (b) MRFB enhanced feature extractor with MRFB; (c) boundary box generator and decoder.

**Figure 8:** P-R curves of different detection models. (a) P-R curves of Cavity; (b) P-R curves of Tree-in-bud pattern.

**Figure 9:** Detection of cavity detection results by YOLOv3 and YOLOv4.

**Figure 10:** Detection of cavity by U-Net, Faster-RCNN and MIP-MY.

**Figure 11:** Detection of the tree-in-bud pattern by YOLOv3 and YOLOv4.

**Figure 12:** Detection of tree-in-bud pattern by U-Net, Faster-RCNN, and MIP-MY.

**Table 1:** The quantitative comparison of performance on each loss function.

Method	mAP (%)	Miss detection rate (%)
*L*_CIOU_	79.47	20
*L*_Class_	78.81	20
*L*_Conf_	76.15	21
*L*_CIOU_ + *L*_Class_	87.41	14
*L*_CIOU_ + *L*_Conf_	85.06	17
*L*_Class_ + *L*_Conf_	84.29	18
Cross-entropy loss	90.36	11
Integrated loss	95.59	6

**Table 2:** The influence of each improved module on the pulmonary *tuberculosis* detection model.

Model	mAP (%)	Parameters (M)	Miss detection rate (%)	Detection time (s)
Model 1	85.86	38.64	16	6.95
Model 2	88.50	39.57	13	7.87
Model 3	91.92	58.29	10	8.86
MIP-MY	95.59	33.91	6	5.88

**Table 3:** Evaluation results of each detection model on test set 2.

Model	Precision (%)	Recall (%)	mAP (%)	Miss detection rate (%)	Parameters (M)	Detection time (s)
U-net [6]	92.20	81.87	88.79	12	96.32	10.36
YOLOv3 [8]	89.14	76.08	74.92	22	61.53	9.63
Faster-RCNN [10]	94.96	83.66	92.40	8	136.65	11.62
YOLOv4 [12]	91.37	81.03	87.21	14	63.94	8.81
MIP-MY	96.59	85.50	95.32	6	33.91	5.72

## Data Availability

The dataset used to support the findings of this study has not been made available because the dataset is provided by the partner hospital and includes patient information.
